# Effect of Steroids on Granulomatous and Non-granulomatous Mastitis: A Case Series of 12 Patients

**DOI:** 10.7759/cureus.92263

**Published:** 2025-09-14

**Authors:** Amog Prakash, Rabbia Khan, Jeyseelan Lakshmanan

**Affiliations:** 1 Internal Medicine, College of Medicine, Mohammed Bin Rashid University of Medicine and Health Sciences, Dubai, ARE; 2 Breast Surgery, Mediclinic, Dubai, ARE; 3 Biostatistics and Epidemiology, Mohammed Bin Rashid University of Medicine and Health Sciences, Dubai, ARE

**Keywords:** breast, cancer, corticosteroids, granulomatous, mastitis

## Abstract

Background and objective: Granulomatous mastitis (GM) is a rare, chronic inflammatory breast condition characterized by granulomatous changes around the lobules and ducts, typically presenting as a unilateral, tender, swollen, and erythematous breast. First described in 1972, its exact cause remains unclear, and there is no standardized first-line treatment. Corticosteroids are commonly used with generally positive outcomes, though they carry risks of side effects and relapse. In a case series of 12 patients with GM-like symptoms, six were confirmed histologically, and all showed improvement with corticosteroids. Diagnosis relies on biopsy, which reveals non-necrotizing granulomas and immune cell infiltration. As GM often mimics bacterial mastitis but is usually sterile, antibiotics are frequently ineffective. In steroid-intolerant or relapsing cases, low-dose methotrexate is a potential alternative, though it has notable side effects.

Materials and methods: For this analysis, patient data from 2022 were retrospectively collected from an electronic medical database, focusing on women aged 18-70 residing in the UAE who presented with breast lumps or pain. Exclusion criteria included pregnancy, male gender, and non-residents of the UAE, as these patients would not be able to attend follow-up consultations to assess treatment effectiveness. Information such as age, marital status, presence of children, presenting symptoms, surgical interventions, medications (antibiotics, steroids, methotrexate, azathioprine), insulin resistance, and biopsy findings were recorded. Biopsies (core needle, excisional, or post-surgical) were reviewed by a pathologist and stained using Ziehl-Neelsen, H&E, and PAS techniques to confirm granulomas. Of 12 patients, six had biopsy-confirmed GM, and 11 were treated with steroids (one opted for observation only). Follow-up included tracking remission, progression, and treatment response. Statistical analysis involved presenting continuous variables such as age as mean ± SD and categorical variables as counts and percentages, with key findings reported with 95% confidence intervals.

Results: This study included 12 married women aged 31 to 45 years (mean age 38.5±4.9 years) treated for granulomatous mastitis. Half (six of 12) had biopsy-confirmed granulomas, while 92% received steroids and 58.3% were treated with methotrexate. Breast abscess was the most common presenting complaint (66.7%), followed by breast mass and mastitis. Co-morbidities were present in 58.3%, with 41.7% showing insulin resistance. All microbiological tests, including cultures and TB screening, were negative. Among the six granuloma-positive patients, five received both steroids and methotrexate. Interestingly, even granuloma-negative patients who received this combination showed similar improvement. One patient who refused steroid treatment continued to relapse. Those treated with steroids showed good clinical and radiological response, with tapering over time. Seven patients who relapsed during steroid tapering were started on methotrexate with low-dose steroids, followed by gradual weaning. All patients responded well and remained symptom-free at six-month follow-up.

Conclusion: This study suggests empiric corticosteroid therapy may be effective for managing recurrent breast inflammation, even without biopsy-confirmed granulomatous mastitis. Both confirmed and suspected cases showed similar outcomes.

## Introduction

Granulomatous mastitis (GM), a rare breast condition that has always been under the scope of research, is a chronic inflammatory condition in which granulomatous change occurs around the lobules and ducts of the breast. Because the condition does not have a specific etiology, there is no approved first-line treatment. Corticosteroids, although very effective, do have their own side effects, adverse reactions, and a high failure rate. Patients typically present with a localized, tender, firm, swollen, and erythematous breast, which is generally unilateral. In this case series, we present 12 patients who presented with the above-mentioned symptoms and were subsequently categorized according to their chief complaint, marital status, co-morbidities, whether they underwent surgical resection, histopathology results, and microbiology findings for any growth. Of the 12, six were proven to have GM on biopsy, which is regarded as the only modality to diagnose this condition, while the others did not show such histological features. However, all of them showed great improvements after starting therapy with corticosteroids.

GM, which was first described in 1972, is a rare chronic inflammatory condition of the breast with an incidence of about 2.4 per 100,000 women and 0.37% in the United States [1]. Because of its rarity, there is still a lack of data on the condition, and a specific first-line therapy does not exist. However, several studies revealed positive effects experienced by patients after using corticosteroids, one of which was well highlighted by Yukawa et al. [2]. Patients typically present with a localized, tender, firm, swollen, erythematous breast, which is generally unilateral [3]. Systemic symptoms such as malaise, fever, and chills have also been reported. Although not very common, palpable reactive axillary lymphadenopathy has also been detected on physical exam [4]. The definitive diagnosis is made using histopathological techniques, which show non-necrotizing granulomas in addition to localized infiltration of multinucleated giant cells, lymphocytes, plasma cells, and epithelioid histiocytes, without cellular atypia. This is usually a diagnosis of exclusion, and management must be tailored according to the symptoms and signs presented [5].

Treatment options widely range from antibiotics, wide surgical excision, abscess drainage, corticosteroids, and even mastectomy, depending on what is most suitable for the patient [6,7]. Since GM often presents with inflammatory breast symptoms, patients are often prescribed antibiotics, which, not surprisingly, fail. GM, in most cases, by definition, is a sterile inflammatory disease [8,9]. Although not well understood, an exaggerated immune response against Corynebacterium has been linked with some cases of GM, which could potentially mimic bacterial mastitis and warrant empirical therapy with antibiotics [10]. Although useful in treatment, several patients were advised to discontinue the drug due to relapse or inability to tolerate it well. In such cases, low-dose methotrexate can be a viable alternative [11]. Adverse effects of methotrexate include ulcerative stomatitis, leukopenia, nausea, abdominal distress, undue fatigue, chills and fever, dizziness, and decreased resistance to infection [12].

With such advancements and current knowledge on the condition, we present 12 patients (all women) who presented with symptoms consistent with mastitis, of whom six were confirmed with GM based on biopsy results, while the rest did not exhibit histological features consistent with GM. However, all of them responded and showed great improvement when treated with a starting dose of corticosteroids (40 mg), while those who did not show such results were placed on 12.5 mg of methotrexate. This poses the question, “Should corticosteroids be prescribed as empirical therapy for patients who present with inflammatory breast conditions?”

## Materials and methods

To carry out the analysis, we first retrospectively collected patient details of those who presented to the clinic during 2022 from the electronic medical database and tabulated them by "patient identifiers," such as age, marital status, presence of offspring, and "clinical data," such as presenting illness, surgical procedure to remove any abscess, administration of empirical antibiotics, steroids, methotrexate, azathioprine, insulin resistance as a co-morbidity, and biopsy findings confirming granulomas.

Inclusion criteria were females aged 18-70 years residing in the United Arab Emirates. Exclusion criteria were pregnant patients, males, and non-residents of the United Arab Emirates. Diagnosis was made by biopsy (core needle biopsy, excisional biopsy, or biopsy of post-surgical specimen) showing non-caseating granulomas, all reviewed by a pathologist. All specimens were examined under Ziehl-Neelsen, H&E, and PAS stains.

The study parameters included the use of methotrexate, the use of steroids, insulin resistance, and whether a biopsy was done. GM is a rare breast condition, with an incidence of 2.4 per 100,000. Due to its rarity, we studied 12 subjects. We identified 12 patients who presented with a lump or pain (mastitis), of whom six showed granulomatous changes on biopsy, while the others did not. However, 11 of the 12 patients were treated with steroids for eight weeks, while one refused treatment and agreed to observation. Follow-up information, such as remission, disease progression, and response to drug therapy, was obtained from clinical appointments and documented accordingly.

For statistical methods, continuous variables such as age were presented as mean and standard deviation, while categorical variables were presented as number and percent, with percentages for important study parameters presented with 95% CI.

Table 1 presents patient information in a structured, tabular format to enhance clarity and organization. The table shows the most common presenting complaints along with the treatments offered and undergone by each patient.

**Table 1:** Patient identifiers and clinical data, including presenting complaint, diagnosis, and drugs administered.

Patient number	Age	Kids	Presenting complaint	Surgical resection	Antibiotics	Culture growth	Tuberculosis	Immunoglobulin G assay	Steroids	Methotrexate	Azathioprine	Insulin resistance
1	43	Yes	Breast abscess	Yes	Yes	No	No	No	Yes	Yes	Yes	Yes
2	31	Yes	Mastitis	No	Yes	No	No	No	Yes	Yes	No	No
3	34	Yes	Breast abscess	Yes	Yes	No	No	No	Yes	Yes	No	Yes
4	36	Yes	Breast abscess	Yes	Yes	No	No	No	Yes	Yes	No	No
5	41	Yes	Breast abscess	No	No	No	No	No	Yes	Yes	No	No
6	36	Yes	Breast abscess	No	No	No	No	No	Yes	Yes	No	Yes
7	31	Yes	Breast abscess	Yes	Yes	No	No	No	Yes	Yes	Yes	No
8	38	Yes	Breast abscess	No	Yes	No	No	No	Yes	No	No	No
9	40	Yes	Breast mass	No	Yes	No	No	No	Yes	No	No	No
10	43	Yes	Breast mass	No	Yes	No	No	No	No	No	No	Yes
11	44	Yes	Mastitis	No	No	No	No	No	Yes	No	No	No
12	45	Yes	Breast abscess	No	Yes	No	No	No	Yes	No	No	Yes

Figure 1 and Figure 2 show the "pre-steroid phase," where the breast ultrasound was taken before steroid administration, and the "post-steroid phase," which shows the breast ultrasound after steroid administration.

**Figure 1:** Breast ultrasound performed in the pre-steroid treatment phase in a patient with recurrent mastitis and persistent breast inflammation, showing increased vascular flow at the 2 o’clock position. Following core biopsy and exclusion of other systemic inflammatory conditions such as sarcoidosis, the patient was started on corticosteroid therapy.

**Figure 2:** A follow-up breast ultrasound performed six weeks after steroid treatment in the same patient demonstrated a favorable response, with almost no vascular markings compared to the image above, and resolution of the inflammatory mass both clinically and radiologically. Histopathological examination revealed no granulomas. The affected area showed significant size reduction, and the patient was managed successfully without antibiotics.

## Results

There were 12 subjects involved in the study. The mean age (standard deviation) of the study subjects was 38.5±4.9 years. The median age was 39 years. The distribution of presenting variables at baseline and at the hospital is shown in Table 1. Table 2 shows the variability among patients with respect to the presenting complaint, investigations performed, and treatments offered and received.

**Table 2:** Distribution of study variables.

Variable	Category	Count	Column, N%
Presenting complaint	Breast abscess	8	66.70%
	Breast mass	2	16.70%
	Mastitis	2	16.70%
Surgical resection	No	8	66.70%
	Yes	4	33.30%
Antibiotic therapy	No	3	25.00%
	Yes	9	75.00%
Culture growth	No	12	100.00%
Tuberculosis	No	12	100.00%
Immunoglobulin G assay	No	12	100.00%
Steroids	No	1	8.30%
	Yes	11	91.70%
Methotrexate	No	5	41.70%
	Yes	7	58.30%
Co-morbidities	No	5	41.70%
	Yes	7	58.30%
Granuloma on biopsy	No	6	50.00%
	Yes	6	50.00%
Azathioprine	No	10	83.30%
	Yes	2	16.70%
Insulin resistance	No	7	58.30%
	Yes	5	41.70%
Granuloma on second biopsy	No	10	83.30%
	Yes	2	16.70%

There were 12 subjects aged 31 to 45 treated for GM included in the study. The mean (SD) age was 38.5±4.9 years. The minimum and maximum ages were 31 and 45 years, respectively. All subjects were married. Six subjects (50%, 95% CI: 21%, 78%) were positive for granuloma biopsy. Steroid use was 92% (76.6%, 100%), and methotrexate use was 58.3% (30.4%, 86.1%). Of the total, eight subjects (66.7%, 40%, 93.3%) had breast abscess. Two subjects each had a breast mass and mastitis. Co-morbidities were present in 58.3% of subjects. Insulin resistance was present in 41.7%, and granuloma positivity on the second biopsy was 2/12 (16.7%). Table 3 shows the proportion of patients with co-morbid insulin resistance who received methotrexate and steroid therapy.

**Table 3:** Distribution of steroids and insulin resistance by methotrexate use.

Variable		Methotrexate			
		No		Yes	
		Count	Row, N%	Count	Row, N%
Steroids	No	1	100.00%	0	0.00%
	Yes	4	36.40%	7	63.60%
Insulin resistance	No	3	42.90%	4	57.10%
	Yes	2	40.00%	3	60.00%
Granuloma on biopsy = no					
Steroids	No	1	100%	0	0.01%
	Yes	3	60.00%	2	40.00%
Granuloma on biopsy = yes					
Steroids	No	0	0.00%	0	0.00%
	Yes	1	16.60%	5	83.40%

Of the six subjects with positive granuloma biopsy, one (16.6%) used steroids, and five (83.4%) did not. Three subjects (60%) negative for granuloma biopsy received steroids. Five (83.4%) subjects positive for granuloma biopsy used both steroids and methotrexate, while two (40%) negative for granuloma biopsy used both. One subject with insulin resistance (8.3%) was granuloma positive. One patient without granulomas refused steroids and continued relapsing with abscess formation. Patients who started steroids were monitored and responded well, with clinical and radiological resolution of symptoms. Steroids were tapered gradually. Seven patients who relapsed during dose reduction started methotrexate; five were granuloma positive and two were not. Both groups showed similar methotrexate response. All seven also restarted low-dose steroids. A maintenance dose of 2.5 mg prednisolone was given for six to eight weeks, while methotrexate was gradually reduced and stopped. Steroids were discontinued after eight weeks. All patients recovered well and remained symptom-free. Clinical and radiological follow-up continued for six months. Table 4 illustrates the recovery outcomes of patients who received steroid therapy compared to those who did not, showing the therapeutic impact of steroids. Of the 11 subjects who received steroids, all (100%) recovered; only one subject who did not receive steroids failed to recover. The association between steroid use and recovery was statistically significant (p<0.01), calculated using Fisher’s Exact Test.

**Table 4:** Recovery of patients who received steroid therapy compared to those who did not.

		Recovery status		Total
		No	Yes	
Steroids	No	1	0	1
	Yes	0	11	11
Total		1	11	12

## Discussion

GM can present in the breast with a wide variety of symptoms, ranging from acute mastitis to high suspicion of malignancy with nodal involvement [13]. Diagnosis in most cases is made only on biopsy [14]. We reviewed our data of such cases presenting with these symptoms; half were found to have granulomas on biopsy, and half had only chronic inflammatory cells. Both groups responded similarly to steroids.

The diagnosis and management of GM can be challenging, and patients may undergo unnecessary surgeries. However, before rushing into any surgical procedure, steroids should be used to assess response. Some clinical situations, however, warrant surgical intervention; for example, a patient presenting with an abscess may require incision and drainage, but excision of inflammatory masses should be avoided [15].

Diagnosis can be made with a core needle biopsy. Whether or not granulomas are present, patients can be safely started on steroids, and response can be assessed clinically and radiologically, with doses adjusted or supplemented with another agent for a short duration. Early recognition and prompt initiation of therapy are key [16].

Our focus was on patients who repeatedly presented with a similar clinical picture of GM but were never found to have granulomas on biopsy and were not diagnosed with other systemic granulomatous diseases. We treated them similarly to GM, and they responded. Chronic inflammatory conditions in the breast were seen in half of our patients with high suspicion of GM, and they responded similarly.

Although this study shows a similar therapeutic response to steroid therapy in patients with and without granulomatous changes on biopsy, large-scale studies are warranted to determine whether steroid therapy can be incorporated into the treatment of breast inflammation, regardless of whether it is granulomatous or non-granulomatous.

One key limitation of this study is the restricted scope for comparative analysis, primarily due to the rarity of the condition. Its low prevalence significantly limits the availability of large, representative sample sizes for robust statistical evaluation. Moreover, the condition is often under-recognized in clinical practice due to a lack of awareness among healthcare professionals and overlap with more common pathologies, such as cutaneous abscesses. This often results in misdiagnosis and repeated use of inappropriate or superficial treatments that do not address the underlying etiology. Consequently, many cases remain undocumented or inaccurately reported, further limiting meaningful comparisons or the establishment of standardized diagnostic and therapeutic protocols.

This study has several important limitations affecting generalizability and interpretability. First, the small sample size of 12 patients limits statistical power and may not capture the full clinical heterogeneity of GM or similar inflammatory breast conditions. The retrospective design introduces risks of selection bias, documentation inconsistencies, and missing data. Moreover, the absence of a defined control group limits the ability to establish causality between corticosteroid therapy and clinical outcomes. Diagnostic uncertainty is another limitation, as only half of the patients had histopathologically confirmed GM, while the others were treated empirically based on clinical suspicion, introducing heterogeneity. Treatment protocols varied across the cohort, with inconsistent use and dosing of corticosteroids, methotrexate, and azathioprine, making it difficult to attribute outcomes to a specific intervention. The relatively short follow-up of six months may not capture long-term outcomes, particularly given the relapsing nature of the condition. The absence of quantitative measures to objectively assess treatment response, such as standardized radiologic or symptom scoring systems, introduces subjectivity. Finally, being a single-center study, these findings may reflect local practices and may not be widely generalizable. These limitations highlight the need for larger, prospective, multicenter trials with standardized diagnostic criteria and treatment protocols to more definitively evaluate corticosteroid therapy in both granulomatous and non-granulomatous inflammatory breast disease.

Short-term steroid therapy, with close clinical and radiological follow-up to assess the size of the inflammatory mass and reactive lymph nodes, will guide physicians on when to taper medication. This can help avoid unnecessary surgical intervention.

## Conclusions

In conclusion, the findings of this study suggest that empirical initiation of corticosteroid therapy may be a safe and effective management strategy for patients presenting with recurrent inflammatory episodes of the non-lactating breast, regardless of histopathological confirmation of GM. The observed clinical and radiological improvement across both granulomatous and non-granulomatous subgroups highlights the potential value of a conservative immunosuppressive approach in avoiding unnecessary surgical interventions, thereby improving patient outcomes and quality of life. Given the diagnostic challenges and variability in clinical presentation, an empiric trial of corticosteroids may serve as both a therapeutic and diagnostic tool in select patients. Nevertheless, the findings should be interpreted with caution due to the limitations of this study, including a small sample size and a lack of standardized treatment protocols. To validate and expand on these preliminary observations, larger-scale, prospective, multi-center studies are warranted. Such studies should incorporate standardized diagnostic algorithms, objective response metrics, and long-term follow-up to better define the role of corticosteroids in managing both confirmed and suspected GM.

## References

[1] Wolfrum A, Kümmel S, Theuerkauf I, Pelz E, Reinisch M (2018). Granulomatous mastitis: a therapeutic and diagnostic challenge. Breast Care (Basel).

[2] Yukawa M, Watatani M, Isono S (2015). Management of granulomatous mastitis: a series of 13 patients who were evaluated for treatment without corticosteroids. Int Surg.

[3] Boakes E, Woods A, Johnson N, Kadoglou N (2018). Breast infection: a review of diagnosis and management practices. Eur J Breast Health.

[4] Mitchell KB, Johnson HM, Rodríguez JM (2022). Academy of breastfeeding medicine clinical protocol. Breastfeed Med.

[5] Özel L, Ünal A, Ünal E (2012). Granulomatous mastitis: is it an autoimmune disease? Diagnostic and therapeutic dilemmas. Surg Today.

[6] Going JJ, Anderson TJ, Wilkinson S, Chetty U (1987). Granulomatous lobular mastitis. J Clin Pathol.

[7] Imoto S, Kitaya T, Kodama T, Hasebe T, Mukai K (1997). Idiopathic granulomatous mastitis: case report and review of the literature. Jpn J Clin Oncol.

[8] Elzahaby IA, Khater A, Fathi A (2016). Etiologic revelation and outcome of the surgical management of idiopathic granulomatous mastitis; an Egyptian centre experience. Breast Dis.

[9] Bashir MU, Ramcharan A, Alothman SB (2017). The enigma of granulomatous mastitis: a series. Breast Dis.

[10] Akbulut S, Arikanoglu Z, Senol A, Sogutcu N, Basbug M, Yeniaras E, Yagmur Y (2011). Is methotrexate an acceptable treatment in the management of idiopathic granulomatous mastitis?. Arch Gynecol Obstet.

[11] Coombe RF, Hamed H (2021). An update on granulomatous mastitis: a rare and complex condition. Br J Hosp Med (Lond).

[12] Tekgöz E, Çolak S, Çinar M, Yilmaz S (2020). Treatment of idiopathic granulomatous mastitis and factors related with disease recurrence. Turk J Med Sci.

[13] Omranipour R, Vasigh M (2020). Mastitis, breast abscess, and granulomatous mastitis. Adv Exp Med Biol.

[14] Yin Y, Liu X, Meng Q, Han X, Zhang H, Lv Y (2022). Idiopathic granulomatous mastitis: etiology, clinical manifestation, diagnosis and treatment. J Invest Surg.

[15] Zhou F, Yu LX, Ma ZB, Yu ZG (2016). Granulomatous lobular mastitis. Chronic Dis Transl Med.

[16] Maung MH, Bethune GC, Patriquin G, Barnes PJ (2020). Cystic neutrophilic granulomatous mastitis - a review of 12 consecutive cases. Histopathology.

